# BrainNet: Optimal Deep Learning Feature Fusion for Brain Tumor Classification

**DOI:** 10.1155/2022/1465173

**Published:** 2022-08-04

**Authors:** Usman Zahid, Imran Ashraf, Muhammad Attique Khan, Majed Alhaisoni, Khawaja M. Yahya, Hany S. Hussein, Hammam Alshazly

**Affiliations:** ^1^Department of Computer Engineering, HITEC University, Taxila 47080, Pakistan; ^2^Department of Computer Science, HITEC University, Taxila, Pakistan; ^3^Computer Sciences Department, College of Computer and Information Sciences, Princess Nourah Bint Abdulrahman University, Riyadh 11671, Saudi Arabia; ^4^Department of Electrical Engineering, Umm Al-Qura University, Makkah, Saudi Arabia; ^5^Electrical Engineering Department, College of Engineering, King Khalid University, Abha 62529, Saudi Arabia; ^6^Electrical Engineering Department, Faculty of Engineering, Aswan University, Aswan 81528, Egypt; ^7^Faculty of Computers and Information, South Valley University, Qena 83523, Egypt

## Abstract

Early detection of brain tumors can save precious human life. This work presents a fully automated design to classify brain tumors. The proposed scheme employs optimal deep learning features for the classification of FLAIR, T1, T2, and T1CE tumors. Initially, we normalized the dataset to pass them to the ResNet101 pretrained model to perform transfer learning for our dataset. This approach results in fine-tuning the ResNet101 model for brain tumor classification. The problem with this approach is the generation of redundant features. These redundant features degrade accuracy and cause computational overhead. To tackle this problem, we find optimal features by utilizing differential evaluation and particle swarm optimization algorithms. The obtained optimal feature vectors are then serially fused to get a single-fused feature vector. PCA is applied to this fused vector to get the final optimized feature vector. This optimized feature vector is fed as input to various classifiers to classify tumors. Performance is analyzed at various stages. Performance results show that the proposed technique achieved a speedup of 25.5x in prediction time on the medium neural network with an accuracy of 94.4%. These results show significant improvement over the state-of-the-art techniques in terms of computational overhead by maintaining approximately the same accuracy.

## 1. Introduction

With the arrival of deep learning (DL), a remarkable change has occurred in the fields related to medical imaging, i.e., magnetic resonance imaging (MRI), computer vision (CV), and many more [1]. A brain tumor is one of the leading causes of death in both males and females. The survival rate of people with a brain tumor is very low, but it can be significantly increased if tumors are detected at an early stage [2]. According to the WHO standard, around 700,000 humans are affected by brain tumors, and since 2019, around 86,000 patients are being diagnosed with this. There have been 16,830 fatalities due to brain tumors since 2019, and the average survival rate is only 35% [3]. In the USA, during 2021, the estimated cases of brain tumors are 83,570 which include 24,530 malignant and 59,040 nonmalignant tumors. The numbers of deaths occurred during 2020 are 18,600. In 2022, the estimated case of brain tumors will be 700,000 in the United States [4].

Tumors are basically malignant cells that are made by the uncontrolled development of the cancerous cells in any part of the body, whereas if this occurs in the brain it results in a brain tumor [5]. There are a lot of medical imaging techniques (MITs) used for the detection of diseases, i.e., computed tomography (CT) [6], magnetic resonance imaging (MRI) [7], ultrasonography [8], and many more [9]. Among all these techniques, magnetic resonance imaging (MRI) is one of the best techniques for the detection of brain tumors [10]. This is because it gives detailed information about the size, type, and position of the cell and is also very sensitive to the local changes in the tissue density [11, 12]. The images gathered from magnetic resonance imagining (MRI) must be analyzed by the experienced neuroradiologist to check for abnormalities within the brain, which requires a lot of time with manual effort. This ends up having a drawback of high cost, due to the need of a highly skilled neuroradiologist, and also because of the time-consuming process [13], so automated procedures are proposed by the researchers.

Automatic detection of brain tumors based on CV has been proposed by most of the researchers [14–16]. These techniques sometimes start with the preprocessing step which is generally used to enhance the image to achieve higher accuracy [17]. However, this is not the obvious case as it depends on the situation whether you need to do the preprocessing or not. As many of the researchers skip this part [18], the images are then used for feature extraction. As we explained earlier in the introduction, DL has shown remarkable results in so many fields, i.e., medical and computer vision (CV). The main problem with the deep learning approach is that it required a large amount of data and very high computational power to train the machine. However, this problem has been solved by the arrival of transfer learning (TL) [19]. In the case of transfer learning, the layers of the pretrained model are generally modified in a way that they can be used for specific problems. Typically, it can be performed by the modification of input and output layers to tune them according to your problem. Most of the researchers used several pretrained deep convolutional neural network (DCNN) models for computer vision and medical imaging, i.e., ResNet [20], Inception-V3 [21], VGG [22], and GoogLeNet [23].

With all this work, there is still a need for a lot more work in the phase of detection and classification. To address these problems, in this article, we proposed an optimal deep learning feature fusion for the classification of brain tumors. Our work is carried out in many steps. However, the main focus of this article is the optimization of deep learning features and after that the fusion of them into one matrix. To summarize, the contribution of our work is as follows:

1. Preprocessing of the dataset (normalization and conversion)
2. Selection of the optimal deep features using two algorithms differential evaluation (DE) and particle swarm intelligence (PSO)
3. Fusion of optimal features by serial fusion to obtain the fused optimal feature vector, which is passed to classifiers for the classification

This article is organized in the following sequence: Section 2 discusses the previous relevant techniques. The proposed work, which includes database creation, selection of an optimal solution, and fusion, is presented in Section 3.  Section 4 presents detailed classification results, and finally, the conclusion of this paper is discussed in Section 5.

## 2. Related Work

Brain tumor classification is an important and hot research topic nowadays. Several techniques have been introduced such as deep learning based, best features selection based, and many more [24–26]. In the literature, in [14], the authors presented an automated system for MRI-based brain tumor images with the help of machine learning techniques. The dataset they used for this is BraTS2017. They carried out this whole process in four steps that are preprocessing, segmentation, feature extraction, and then classification. Initially, in the preprocessing phase, they manually removed the skull and reduced the noise with the help of the median filter. In the segmentation, they used Chan–Vese (CV), and then, the features were extracted with the help of a gray-level co-occurrence matrix (GLCM). They used two classifiers SVM and KNN that are used for the performance evaluation, which outperformed the existing methods. They achieved an accuracy of about 98.13% for the SVM and 92.30% for the KNN.

A computer-aided diagnosis (CAD) system has been proposed in [26]. To achieve promising experimental evaluation for two different types of datasets, a recognition scheme named multi-level attention network (MANet) that is both cross-channel and spatial attention was proposed. The evaluated datasets are BraTS2018 and Figshare. The experimental result shows that this CAD technique achieved an accuracy of 94.91% on BraTS2018 and 96.51% on Figshare. Another novel computer-aided diagnosis (CAD) technique is presented in [27]. This technique extracts the features with the help of discrete wavelet transform (DFT). Later, these extracted features are then passed to the CNN to classify the input MRI images. In the experimental process, they achieved an accuracy of 99.3%.

A deep learning approach is presented in [18] to classify brain tumor disease. The datasets they used for this were BraTS2018 and BraTS2019. To extract the features, they utilized transfer learning to fine-tune the Densenet201 model. Later, they applied the entropy-kurtosis-based high feature value (EKbHFV) and the modified genetic algorithm (MGA) to select the optimal features. Fusion is performed with the help of a nonredundant serial-based approach and then classified by the cubic SVM. They achieved an accuracy of more than 95%. The authors of [17] examine the performance of multiple deep learning models, i.e., VGG16, AlexNet, GoogleNet, and ResNet50, in terms of their ability to examine the brain tumor. For evaluation, they used the criteria of accuracy and processing time. The result shows that ResNet50 gave the highest accuracy of about 95.8%, and AlexNet has the fast processing of about 1.2 sec which then decreases to 8.3 msec using GPU.

Brain tumor classification by the combination of both machine learning and deep learning approaches is presented in [28]. They used three different brain tumor classes named glioma, meningioma, and pituitary for classification. To extract the deep features, they utilized transfer learning to fine-tune the GoogLeNet model. The extracted features are then classified with the help of the support vector machine (SVM), K-nearest neighbor (KNN), and softmax.

A computer-aided approach is presented in [16] to classify the brain MRI images. The author considered two classes that are the normal class and tumor class. The proposed technique was named 2D convolution neural network. The evaluation results are compared based on the recall value, *F*1-score value, and precision value. Their proposed method gave an accuracy of 97%.

In [29], H. A. Khan et al. presented a convolutional neural network (CNN) model for the classification of the brain tumor along with augmentation and image processing. Initially, in the image processing phase, they used canny edge detection to crop the black portion from an image. After this, they performed the data augmentation to increase the number of images in the dataset. They performed the augmentation by making minor changes in images like rotation, brightness, and flipping. Then, they compared their proposed convolution neural network (CNN) model with the pretrained VGG-16, ResNet-50, and Inception-V3 models. The experimental results were evaluated on very small data which gave the accuracy of about 100%, 96%, 89%, and 75% for their proposed CNN, VGG-16, ResNet-50, and Inception-V3, respectively.

In conclusion, the strategies discussed above primarily aimed to strengthen the extracted features in order to improve the outcome of the presented techniques. They also demonstrated the significance of classifiers in improving classification accuracy. In the classification phase, the failure to extract the best features and the problem of overfitting are the fundamental shortcomings of these strategies. We focused on the fusion of features for brain tumor categorization in this paper. We concentrated on extracting useful deep learning characteristics. Furthermore, we focused on the problem related to overfitting and then feature selection, with the goal of reducing prediction time without sacrificing too much on the accuracy. We proposed an end-to-end automated technique to address these gaps.

## 3. Proposed Methodology

We present a fully automated technique for brain tumor classification in this paper. This study looks at four different types of brain tumors. The following are the steps involved in this implementation:

1. Preprocessing is applied to normalize the dataset and convert images from single to multichannel (requirement of the deep learning model).
2. The ResNet101 pretrained model is fine-tuned using the transfer learning technique in order to use it for disease classification.
3. The DE and PSO algorithms are used to calculate two optimized feature vectors.
4. Using the serial fusion technique, we combine the two feature vectors to get the fused feature vector.
5. We apply PCA to the fused vector in order to select the top high variance features.
6. Different classifiers are used to classify these features.  Figure 1 shows the block diagram of the proposed approach.

### 3.1. Database Preparation

In this paper, BraTS2018 is used for evaluation purpose. This dataset is clinically acquired preoperative multimodal MRI scans of glioblastoma (GBM/HGG) [30]. This dataset is divided into four categories: (a) native (**T1**), (b) postcontrast T1-weighted (**T1CE**), (c) T2-weighted (**T2**), and (d) T2 fluid-attenuated inversion recovery (**FLAIR**). T1 is composed of 28,446 images, T1CE is composed of 28,969 images, T2 is composed of 28,759 images, and FLAIR is composed of 28,413 images. These images are all in grayscale format with a resolution of 240 × 240 pixels.  Figure 2 shows a few examples of images.  Table 1 provides a summary of the overall images.

### 3.2. Resnet101 Deep Model

Deep neural networks have made significant progress in the field of image classification in recent years. A deep model, by definition, is the combination of low-level, mid-level, and high-level features, as well as a classifier. We used ResNet101 [31] to extract deep features in this paper. The VGG19 pretrained network, which is one of the deepest convolutional neural networks (CNNs), inspired this architecture. A CNN model, as previously stated, is made up of many different layers that are connected to each other. These layers are used for a variety of tasks, such as natural language processing and medical image classification. The convolutional filter size in ResNet101 is 33, and the stride value is 2. Downsampling is performed in the convolutional layers based on the stride value. This network has 347 layers and 379 connections. The input to the network has a dimension of 224 × 224 × 3. The filter size is [7, 7], the number of channels is 3, and the number of filters is 64 in the first convolution layer. The filter size in the max pooling layers is 3 × 3, and the stride value is 2. The number of channels and filters in the second convolutional layer is 64. The number of filters in the final convolution layer is 2048, with 512 channels [32]. We get an output vector of dimension *N* × 2048, where N denotes the number of features, by extracting features from the pool5 layer.  Figure 3 depicts the ResNet101 architecture in its entirety.

### 3.3. Transfer Learning-Based Network Training

In deep learning, data reliance is a severe issue. In comparison to typical machine learning techniques, a large amount of data is needed to train a deep model. The fundamental reason for this enormous amount of training data is that it is necessary to learn hidden patterns. However, a large amount of data is not often accessible for training a deep learning model in a few study domains, particularly in medical imaging. The concept of transfer learning (TL) [33] is to train a model with less data. It is not necessary to train the target model from scratch in TL. Deep transfer learning is defined mathematically as follows.

Given a transfer learning task with the following parameters: 〈*D*_*s*_, *T*_*s*_, *D*_*t*_, *T*_*t*_, *F*_*t*_(·)〉, *D*_s_ represents the source domain, *T*_s_ and *T*_t_ represent the learning task from the source and the target, *D*_t_ represents the target domain, and *F*_t_ (.) represents the nonlinear function that represents a deep neural network.  Figure 4 depicts the model learning process using transfer learning graphically. In this figure, it is shown that the original ResNet101 model is trained on the ImageNet dataset [34], and then, knowledge is transferred using deep transfer learning for retraining this model on the target database. As a target database, the brain tumor database is used. We extract features from the pool5 layer and output a vector of dimension *N* × 2048. We started with a learning rate of 0.0001 and a minimum batch size of 32 in the learning.

#### 3.3.1. Training Process

Figure 5 depicts the deep learning model's complete training procedure. The following is a description of the figure.

1. We divide each class such as T1, T1CE, T2, and FLAIR into 50% training and testing images. A randomized procedure is used to separate these images.
2. The ResNet101 model was trained using deep transfer learning for brain tumor classification.
3. Deep learning features are extracted from the pool5 layer.
4. DE and PSO are two optimization strategies that are used to improve the extracted features.
5. As the output, two optimal feature vectors are returned.
6. We perform fusion of both optimal vectors using serial fusion.
7. We apply PCA to the fused vector.
8. We train the classifier and save the model for testing.

We train and save our model for brain tumor categorization based on the aforementioned methods. The following sections go over the optimization, fusion, PCA, and classification stages in detail.

### 3.4. Feature Optimization

The classification accuracy is improved by selecting the most optimal set of features from the initial set of features. These features were chosen for learning from original features with the least amount of loss. The main advantages are that they improve accuracy, take less time, and eliminate the issue of overfitting. In feature selection, the optimization process entails determining the optimum feasible values depending on the established objective function. Many evolutionary strategies for identifying the closest optimal solution are provided for this aim. We implemented two algorithms in this article: differential evolution (DE) and particle swarm intelligence (PSO).

#### 3.4.1. Differential Evolution

The DE is a global search optimization problem-solving evolutionary approach [35]. Because it uses fewer control factors than the genetic approach (GA), this technique is easier to use. It is significantly more effective in the realm of medical imaging because it has fewer control factors. It starts with a set of randomly generated starting values in the search space. The input data are then subjected to mutation and crossover, followed by a selection procedure to establish a new population. The steps involved in this project are listed as follows:

**Input:** original *N* × 2048 dimensional deep feature vector.

**Output:** optimal feature vector of dimension *N* × 1119.

(1) Step 1: We initialize the following parameters:
  (1) Population = 50
  (2) Minimum bound and maximum bound
  (3) Use the following expression to find these bounds:
    (1) $$\begin{array}{c} \lambda_{i}^{j}=\lambda_{\text{min}}^{j}+\text{rand}\left(0,1\right)\cdot \left(\lambda_{\text{max}}^{j}-\lambda_{\text{min}}^{j}\right). \end{array}$$
(2) Step 2: We calculate the fitness function, where fine KNN is opted as the fitness function, and the mean square error rate (MSER) is used for the performance evaluation.
(3) Step 3: We perform mutation as shown in the following equation:
  (2) $$\begin{array}{c} M_{r}=0.2. \end{array}$$
(4) The following equation is used to define mutation:
  (3) $$\begin{array}{c} \nu_{i}^{j}=\lambda_{r_{1}}^{j}+F\left(\lambda_{r_{2}}^{j}-\lambda_{r_{3}}^{j}\right). \end{array}$$
(5) Step 4: We perform crossover as shown in the following equation:
  (4) $$\begin{array}{c} C_{r}=0.7,\\ C_{i}^{j}=\left\{\nu_{i}^{j},\;\text{if rand}\left(0,1\right)\leq C_{r}\text{ or }j=j_{\text{rand}}\lambda_{i}^{j},\text{ Otherwise}\right.. \end{array}$$
(6) Step 5: We find fitness evaluation and selection. We repeat steps 2, 3, and 4 until the required optimal feature vector is obtained. An optimal feature vector of dimension *N* × 1119 is obtained as a result.

#### 3.4.2. Particle Swarm Optimization

Particle Swarm Optimization (PSO) is inspired by swarm behavior such as bird flocks and schooling fish. PSO is basically a population-based metaheuristic technique [36]. It is an efficient evolutionary algorithm, that is why it is extensively used to solve single or multiple-objective problems [37]. Furthermore, PSO is also a powerful computing tool in terms of speed and memory usage [38].

Particle Swarm Optimization (PSO) works on the basis of 5 steps that are mentioned as follows:

**Input:** original *N* × 2048 dimensional deep feature vector.

**Output:** optimal feature vector of dimension *N* × 1125.

(1) Step 1: We perform generation of population as shown in the following equation:
  (5) $$\begin{array}{c} \text{Population}=p_{\text{gen}}\left(\text{gen}=0,1,\ldots ,{\text{Max}}_{\text{gen}}\right)\\ p=\left[\begin{array}{ccccc} b_{11}^{L} & b_{12}^{L} & b_{13}^{L} & \ldots & b_{1M}^{L}\\ b_{21}^{L} & b_{22}^{L} & b_{23}^{L} & \ldots & b_{2M}^{L}\\ \ldots & \ldots & \ldots & \ldots & \ldots \\ b_{N1}^{L} & b_{N2}^{L} & b_{N3}^{L} & \ldots & b_{NM}^{L} \end{array}\right], \end{array}$$
  where *b*_11_^*L*^ *b*_12_^*L*^ *b*_13_^*L*^ … …*b*_1*M*_^*L*^ denotes the particle/candidate solution. Single individual, i.e., *b*_11_^*L*^ called as an agent. “P” basically denotes the population.
(2) Step 2: We calculate the fitness function, where fine KNN is opted as the fitness function, and the mean square error rate (MSER) is used for the performance evaluation.
(3) Step 3 (a): We find the local best. We find the local best from the first candidate solution
  (6) $$\begin{array}{c} C=b_{11}^{L}b_{12}^{L}b_{13}^{L}\ldots \ldots b_{1M}^{L}, \end{array}$$
  where *C* is the first candidate solution,
  (1) *lb*=*C*_1_
  (2) ∀*i*=2 to *L*
  (3) if fitness(*C*_*i*_) > fitness(*lb*)
  (4) then
  (5) *lb*^*i*^=*C*_*i*_
  (6) else
  (7) continue
  (8) end
(4) Step 3 (b): We find the global best with the help of the following steps:
  (1) To find the global best
  (2) *gb*=*lb*_1_
  (3) ∀*k*=1 to *N*
  (4) if fitness(*lb*_*k*_) > fitness(*gb*)
  (5) then
  (6) *gb*=*lb*_*k*_
  (7) else
  (8) continue
  (9) end
(5) Step 4: We update the speed and position. The equation to update the speed is
  (7) $$\begin{array}{c} V_{n+1}=\omega V_{3}+C_{1}\text{ rand}\left(lb-b_{i}\right)+C_{2}\text{rand}\left(gb-b_{i}\right), \end{array}$$
  where *V*_3_ is the old speed, *C*_1_ and *C*_2_ are the controlling parameters, *ω* is the inertia, (*lb* − *b*_*i*_) is the local updation, (*gb* − *b*_*i*_) is the global updation, *C*_1_ rand(*lb* − *b*_*i*_) is the local intelligence, and *C*_2_ rand (*gb* − *b*_*i*_) is the global intelligence. All these parameters are combined to generate the updated speed which is *V*_*n*+1_.
(6) The equation to update the position is
  (8) $$\begin{array}{c} X_{n+1}=X_{n}+V_{n+1}, \end{array}$$
  where *X*_*n*_ is the old position and *V*_*n*+1_ is the updated speed. By the combination of these parameters, we achieved the updated position.
(7) Step 5: We find fitness evaluation and selection and repeat steps 2, 3, and 4 until the required optimal feature vector is obtained. In the output, an optimal feature vector of dimension *N* × 1125 is obtained.

### 3.5. Feature Fusion

Feature fusion is a process in which two feature vectors are combined to get one feature vector, which is more appealing and discriminating than the two input feature vectors.

One of the biggest advantages of feature fusion is that it improves the image information in terms of features. In this paper, we implement the serial-based extended (SBE) approach for feature fusion.

Following are the two optimal feature vectors denoted by FV_(DE)_^*k*_1_^ and FV_(PSO)_^*k*_2_^ with the length of *N* × 1119 and *N* × 1125, respectively. Let FV_(*fus*)_^*k*^ be the fused feature vector with the dimension of *N* × *K*, where *k* is basically the length of the feature vector after the fusion. Let ‘Y' be the number of features of DE and ‘Z' be the number of features of the PSO, then serial fused features ‘K' have (*Y* + *Z*) dimensions.

The fusion process includes the following steps:

1. Input both optimal feature vectors
2. The size of these vectors is *N* × 1119_DE_ and *N* × 1125_PSO_
3. A final resulting fused feature vector of dimension (DE + PSO) *N* × 2244 is obtained in the output

At last, the fused vector is fed into the different classifiers, which produces two outputs: labeled prediction results and numerical results.  Figure 6 depicts the labeled results, whereas Section 4 has the numerical results.

### 3.6. Principal Component Analysis

PCA (principal component analysis) is a dimensionality reduction technique [39]. This technique is normally carried out to reduce the dimensionality of huge data/feature vectors. This is performed because smaller data are easier to understand and analyze, and machine learning and deep learning algorithms can interpret them much more efficiently and rapidly [40]. PCA keeps only those features that carry a massive amount of information. This is accomplished by preserving just those components that have high variance [41].

Following is the optimal feature vector obtained by the optimal feature fusion denoted by FV_(FUS)_ with the dimension of *N* × 2244. We passed this feature vector to the PCA. The high variance features which we have selected from this are of dimension *N* × 1000. The detailed discussion about the accuracy achieved and the prediction time speedup is discussed below in the result section.

## 4. Results and Discussion

This section covers the detailed discussion about the numerical results we obtained for this work.

The dataset that we used for our experiments is ‘BraTS2018'. This dataset is clinically acquired preoperative multimodal MRI scans of glioblastoma (GBM/HGG) [30]. Originally, this dataset consists of 130,200 images with 4 classes that are (a) native (**T1**), (b) postcontrast T1-weighted (**T1CE**), (c) T2-weighted (**T2**), and (d) T2 fluid-attenuated inversion recovery (**FLAIR**). Most of the images in the given dataset are totally black without any information in them.

In the preprocessing phase, we cleaned the dataset by removing the blank images. After the preprocessing, we ended up having 114,587 images, which we used for the training purpose. We computed the results in multiple steps: (a) with the help of a pretrained deep learning model, we extracted the deep features, and then, we obtained the accuracy by passing them to the different classifiers; (b) to select the optimal feature selection, we first used the differential evolution (DE); (c) then, we used the particle swarm optimization (PSO) and evaluated the results; (d) we fused both of these optimal feature vectors; (e) we compared the results. In the training testing phase, 10-fold cross-validation is used.

Multiple classifiers are utilized in order to compare the accuracies. These classifiers are the fine tree, linear discriminant, cubic SVM, boosted tree, bagged tree, subspace discriminant, narrow neural network, medium neural network, and wide neural network. Various performance metrics are used to report the results, such as the accuracy (%), prediction time (sec), sensitivity, precision, FPR, FNR, and area under curve.

The hyper parameters that we used for our work were as follows:

1. Epochs = 100
2. Learning rate = 0.05
3. Optimizer = stochastic gradient descent
4. Loss function = cross entropy
5. Momentum = 0.7

In order to conduct our experiments, we used Intel Core-i7 6th generation with 16 GB RAM and Nvidia GeForce GTX1070 GPU with 8 GB RAM. We used Matlab 2021a for our simulations.

This section contains the numerical results that we obtained from our experiments. Prediction accuracy of brain tumor disease with the help of original ResNet deep features is presented in Table 2. Among all the classifiers, the cubic SVM gives the highest accuracy of about 96.7%. The negative rate of cubic SVM is 3.3% with a prediction time of 4461.8 seconds. The wide neural network gives the second highest accuracy of about 96.1%. The negative rate of the WNN is 3.9% with a prediction time of 1310.4 seconds. The medium neural network gives the third highest accuracy of about 96%. The negative rate of the MNN is 4% with a prediction time of 4906.5 seconds. The prediction time of brain tumor disease with the help of original ResNet deep features is presented in Table 3. Based on the prediction time, the fine tree is executed in the minimum time of 286.34 seconds. The linear discriminant is the second and the bagged tree is the third best classifier with a minimum prediction time of 336.99 and 774.26 seconds, respectively. The accuracies of these classifiers are 7.1%, 0.7%, and 1.2% with a less difference of 4175.46, 4124.81, and 3687.54 seconds, respectively, in the prediction time as compared to the cubic SVM. The confusion matrix of the cubic SVM on original features is also shown in Figure 7.

Results gathered after the optimal feature selection by PSO are shown in Table 2. Of all the classifiers, the cubic SVM gives the highest accuracy of about 96.7%. The negative rate of the cubic SVM is 3.3% with a prediction time of 954.87 seconds. The negative rate of the cubic SVM by PSO is the same as that of the original one with a decrease of 3506.93 seconds in the prediction time. The wide neural network gives the second highest accuracy of about 95.9%. The negative rate of this classifier is 4.1% with a prediction time of 404.63 seconds. In the case of the wide neural network by PSO, the negative rate is increased by only 0.2% than that of the original one with a decrease of 905.77 seconds in the prediction time. The medium neural network gives the third highest accuracy of about 95.8%. The negative rate of this classifier is 4.2% with a prediction time of 1457.7 seconds. In the case of the medium neural network by PSO, the negative rate is increased by only 0.2% than that of the original one with a decrease of 3448.8 seconds in the prediction time. The prediction time of brain tumor disease with the help of PSO is presented in Table 3. Comparison based on time shows that the linear discriminant will be executed in the minimum time of 62.48 seconds. The fine tree is the second and bagged tree is the third best classifier with a minimum prediction time of 139.28 and 326.44 seconds, respectively. The accuracies of these classifiers are 1%, 7.9%, and 1.3% with a less difference of 892.39, 815.59, and 628.43 seconds, respectively in the prediction time as compared to the cubic SVM. The confusion matrix of the cubic SVM after PSO is also shown in Figure 8.

Results gathered after the optimal feature selection by DE are shown in Table 2. Of all the classifiers, the cubic SVM gives the highest accuracy of about 96.6%. The negative rate of the cubic SVM is 3.4% with a prediction time of 2088.8 seconds. The negative rate of the cubic SVM by DE is increased by only 0.1% than that of the original one with a decrease of 2373 seconds in the prediction time. The wide neural network gives the second highest accuracy of about 96.1%. The negative rate of this classifier is 3.9% with a prediction time of 701.48 seconds. The negative rate of the wide neural network by DE is the same as that of the original one with a decrease of 608.92 seconds in the prediction time. The medium neural network gives the third highest accuracy of about 95.8%. The negative rate of this classifier is 4.2% with a prediction time of 3636.3 seconds. In the case of the medium neural network by DE, the negative rate is increased by only 0.2% than that of the original one with a decrease of 1270.2 seconds in the prediction time. The prediction time of brain tumor disease with the help of DE is presented in Table 3. Now, if we compare this in terms of time, then the linear discriminant will be executed in the minimum time of 117.11 seconds. The fine tree is the second and the bagged tree is the third best classifier with a minimum prediction time of 159.25 and 460.75 seconds, respectively. The accuracies of these classifiers are 1%, 8.6%, and 1.3% with a less difference of 1971.69, 1929.55, and 1628.05 seconds, respectively, in the prediction time as compared to the cubic SVM. The confusion matrix of the cubic SVM after DE is also shown in Figure 9.

Results gathered after the PSO and DE feature fusion are shown in Table 2. Of all the classifiers, the cubic SVM gives the highest accuracy of about 96.7%. The negative rate of the cubic SVM is 3.3% with a prediction time of 3901.4 seconds. The negative rate of the cubic SVM by fusion is the same as that of the original one with a decrease of 560.4 seconds in the prediction time. The linear discriminant gives the second highest accuracy of about 95.7%. The negative rate of this classifier is 4.3% with a prediction time of 52.093 seconds. In the case of the linear discriminant by fusion, the negative rate is only increased by only 0.3% than that of the original one with a decrease of 284.897 seconds in the prediction time. The wide neural network and the subspace discriminant give the third highest accuracy of about 95.4%. The negative rates of these classifiers are 4.6% with a prediction time of 100.38 and 552.78 seconds, respectively. In the case of the wide neural network and the subspace discriminant by fusion, the negative rate is increased by only 0.7% and 0.4%, respectively, than that of the original one with a decrease of 1210.02 and 2510.42 seconds, respectively, in the prediction time. The prediction time of brain tumor disease with the help of feature fusion is presented in Table 3. Now, if we compare this in terms of time, then the linear discriminant will be executed in the minimum time of 52.093 seconds. The wide neural network is the second and the fine tree is the third best classifier with a minimum prediction time of 100.38 and 156.73 seconds, respectively. The accuracies of these classifiers are 1%, 1.3%, and 4.1% with a less difference of 3849.307, 3801.02, and 3744.67 seconds, respectively, in the prediction time as compared to the cubic SVM. The confusion matrix of the cubic SVM after feature fusion is also shown in Figure 10.

Table 2 also shows the percentage difference between the original and fused features. This is also shown visually in Figure 11. The cubic SVM shows the same accuracy after fusion as that of the original one. The accuracy of the fine tree is increased by around 3.3%.

In case of the linear discriminant and the boosted tree, the decrease in the accuracy is only about 0.3%.

The accuracy of the subspace discriminant, wide neural network, bagged tree, medium neural network, and narrow neural network is decreased by around 0.4%, 0.7%, 1%, 1.7%, and 1.9%, respectively. From the results, it is clear that the accuracy remains the same. However, we come up with a decrease in the prediction time as compared to that of the original one, which we will explain later in Table 3 explanation.

Table 3 also shows the speedup between the original and fused features. This is also shown visually in Figure 12. The highest speedup which we achieved is about 25.5 times in the case of the medium neural network. In the case of the wide neural network, the speedup is 13.1 times. The speedup of 6.5, 5.5, and 3.6 times is achieved in the case of the linear discriminant, subspace discriminant, and narrow neural network. In the case of the boosted tree, bagged tree, fine tree, and cubic SVM, we achieved a speedup of 2.1x, 1.9x, 1.8x, and 1.1x, respectively.

Apart from the accuracy and prediction time results presented in Tables 2 and 3, respectively, we also report the detailed results after future fusion. These results are provided in Table 4 where sensitivity, FNR, precision, FPR, and AUC results are provided for various classifiers. All the classifiers have a good performance on all these metrics.

Finally, we also compare our results with the state-of-the-art techniques performing brain tumor classification on the BraTS2018 dataset. This comparison is provided in Table 5. Column 2 shows that the proposed technique has the highest accuracy as compared to the other techniques. Though this improvement in accuracy is not very high, if we bring execution time into the picture (Column 3), we can see that most of the work did not focus on this aspect and did not report it. Our work achieved an improvement of about 25.5x, which is a significant reduction in the prediction time.

## 5. Conclusion

The manual procedure of brain tumor detection and classification is not a good choice as it is tedious, time consuming, and expensive. A fully automated optimal deep feature fusion-based architecture is proposed in this work for brain tumor classification. A database of MRI images is prepared which consists of four different categories of tumors to perform evaluation. The proposed method achieved an accuracy of about 96.7%, which is the highest compared to the existing techniques. Based on the results presented in this work, it is observed that a few redundant and irrelevant features were still perceived. Therefore, it is essential to select the optimal features. It is also shown that the fusion of optimal features improved the accuracy, but reduction in the prediction time is quite significant, obtaining the main goal of this work. The major dark side of this work is the fusion process that increases the computational time during the testing process. In the future, lightweight deep learning frameworks will be opted, and we will utilize an optimized feature fusion approach for classification and detection of tumors [45–49].

## Figures and Tables

**Figure 1:** The proposed approach for the brain tumor classification.

**Figure 2:** Sample database images.

**Figure 3:** ResNet101 architecture.

**Figure 4:** Deep transfer learning process.

**Figure 5:** The proposed training process of the deep learning model for brain tumor classification.

**Figure 6:** Prediction results in the form of labeled Images (a) numerical results.

**Figure 7:** The confusion matrix of the cubic SVM after the original feature classification.

**Figure 8:** The confusion matrix of the cubic SVM after applying the particle swarm optimization (PSO)-based feature selection.

**Figure 9:** The confusion matrix of the cubic SVM after applying the differential evolution (DE)-based feature selection.

**Figure 10:** The confusion matrix of the cubic SVM after applying the optimal feature fusion.

**Figure 11:** Comparison of accuracy results with state of the art.

**Figure 12:** Comparison of the prediction time (logarithmic scale) with state of the art.

**Table 1:** Summary of the dataset.

Class	Database name	Total images
T1	BraTS2018	28,446
T1CE		28,969
T2		28,759
FLAIR		28,413

**Table 2:** Comparison of prediction accuracy of brain tumors.

Accuracies %					
Classifiers	Org. ResNet101	Optimized		Feature fusion	%Age difference (org VS FF)
		PSO	DE		
Fine tree	89.6	88.8	88	92.6	3.3%
Linear discriminant	96	95.7	95.6	95.7	−0.3%
Cubic SVM	96.7	96.7	96.6	96.7	0%
Boosted trees	92.8	92.1	92.3	92.5	−0.3%
Bagged trees	95.5	95.4	95.3	94.5	−1%
Subspace discriminant	95.8	95.5	95.4	95.4	−0.4%
Narrow neural network	95.7	95.5	95.4	93.9	−1.9%
Medium neural network	96	95.8	95.8	94.4	−1.7%
Wide neural network	96.1	95.9	96.1	95.4	−0.7%

**Table 3:** Comparison of the prediction time (sec) of brain tumors.

Prediction time (sec)					
Classifiers	Original ResNet101	Optimized		Feature fusion	Speedup (org VS FF)
		PSO	DE		
Fine tree	286.34	139.28	159.25	156.73	1.8x
Linear discriminant	336.99	62.48	117.11	52.093	6.5x
Cubic SVM	4461.8	954.87	2088.8	3901.4	1.1x
Boosted trees	5615.4	2691.4	3013.2	2688.8	2.1x
Bagged trees	774.26	326.44	460.75	403.45	1.9x
Subspace discriminant	3063.2	688.63	1287.2	552.78	5.5x
Narrow neural network	5999.1	1332.7	2754.2	1662.1	3.6x
Medium neural network	4906.5	1457.7	3636.3	192.56	25.5x
Wide neural network	1310.4	404.63	701.48	100.38	13.1x

**Table 4:** Detailed result after feature fusion.

Fusion detail results					
Classifiers	Sensitivity	FNR	Precision	FPR	AUC
Fine tree	92.575	7.425	92.575	0.0275	0.925
Linear discriminant	95.7	4.3	95.775	0.0125	0.9575
Cubic SVM	96.75	3.25	96.75	0.01	0.97
Boosted trees	92.5	7.5	92.8	0.0225	0.925
Bagged tree	94.475	5.525	94.55	0.02	0.945
Subspace discriminant	95.45	4.55	95.45	0.015	0.9525
Narrow neural network	93.9	6.1	93.9	0.02	0.94
Medium neural network	94.425	5.575	94.425	0.02	0.9425
Wide neural network	95.375	4.625	95.375	0.015	0.955

**Table 5:** A comparative study of the proposed methodologies on the BraTS2018 dataset.

Research papers	Maximum achieved accuracy (%)	Maximum achieved execution-time speedup
PSO features + softmax [42]	92.50	NA
PLS features + ELM [43]	93.40	NA
Two-channel DNN [44]	93.69	NA
MANet [26]	94.91	NA
**Proposed**	**96.7**	**25.5x**

Bold represents the best values.

## Data Availability

The BraTs2018 dataset has been used in this work for the experimental process (http://www.med.upenn.edu/sbia/brats2018/data.html).
